The article "Changes in depression and suicidal ideation under severe lockdown restrictions during the first wave of the COVID-19 pandemic in Spain: a longitudinal study in the general population" was retracted in 2023. Reasons: errors in the data; errors in the analysis; errors in the methods; errors in the results or conclusions.

# Changes in depression and suicidal ideation under severe lockdown restrictions during the first wave of the COVID-19 pandemic in Spain: a longitudinal study in the general population

**DOI:** 10.1017/S2045796021000408

**Published:** 2021-06-02

**Authors:** J. L. Ayuso-Mateos, D. Morillo, J. M. Haro, B. Olaya, E. Lara, M. Miret

**Affiliations:** 1 Department of Psychiatry, Hospital Universitario de La Princesa, Instituto de Investigación Sanitaria Princesa (IIS-Princesa), Madrid, Spain; 2 Instituto de Salud Carlos III, Centro de Investigación Biomédica en Red de Salud Mental, CIBERSAM, Madrid, Spain; 3 Department of Psychiatry, Universidad Autónoma de Madrid, Madrid, Spain; 4 Parc Sanitari Sant Joan de Déu, Universitat de Barcelona, Sant Boi de Llobregat, Barcelona, Spain

**Keywords:** Depression, population survey, risk factors, suicide

## Abstract

**Aims:**

To assess whether there is a change in the prevalence of depression and suicidal ideation after the strict lockdown measures due to the first wave of the COVID-19 pandemic in Spain; and to assess which are the factors associated with the incidence of a depressive episode or suicidal ideation during the lockdown.

**Methods:**

Data from a longitudinal adult population-based cohort from the provinces of Madrid and Barcelona were analysed (*n* = 1103). Structured face-to-face home-based interviews (pre-pandemic) and telephone interviews were performed. Both depression and suicidal ideation were assessed through an adaptation of the Composite International Diagnostic Interview (CIDI 3.0). A variety of validated instruments and sociodemographic variables including age, sex, educational level, occupational status, home quietness, screen time, resilience, loneliness, social support, physical activity, disability, economic situation and COVID-19-related information were also considered. Population prevalence estimates and multivariable logistic regressions were computed.

**Results:**

Overall, prevalence rates of depression and suicidal ideation did not change significantly from before to after the COVID-19 outbreak. However, the rates of depression among individuals aged 50+ years showed a significant decrease compared to before the pandemic (from 8.48 to 6.41%; *p* = 0.01). Younger individuals (odds ratio (OR) = 0.97 per year older; 95% confidence interval (CI) = 0.95–0.99) and those feeling loneliness (OR = 1.96; 95% CI = 1.42–2.70) during the lockdown were at an increased risk of developing depression during the confinement. Resilience showed a protective effect against the risk of depression (OR = 0.46; 95% CI = 0.32–0.66) and suicidal ideation (OR = 0.33; 95% CI = 0.16–0.68), whereas individuals perceiving social support were at a lower risk of developing suicidal thoughts (OR = 0.35; 95% CI = 0.18–0.69).

**Conclusions:**

Continuous reinforcement of mental health preventive and intervening measures during and in the aftermath of the crisis is of global importance, particularly among vulnerable groups who are experiencing the most distress. Future research should strive to evaluate the long-term effects of the COVID-19 crisis on mental health.

## Introduction

The COVID-19 outbreak and the policies to prevent its spread have disrupted the daily living of the population. The evidence regarding the mental health consequences of the confinement due to the COVID-19 pandemic in the general population is inconclusive (O'Connor *et al*., 2020; Bueno-Notivol *et al*., 2021; Faust *et al*., 2021; Prati and Mancini, 2021; Tanaka and Okamoto, 2021; van der Velden *et al*., 2021).

The lockdown in Spain was one of the most restrictive in Europe (García-Esquinas *et al*., 2021). The Government imposed a State of Alarm starting on 15th March that established a national lockdown that included the imposition of distancing measures such as the closure of non-essential customer-facing businesses and educational institutions (Real Decreto, 463/2020). In order to avoid the saturation of the intensive care units, theses initial measures were strengthened with another decree from the Government on 29th March (Real Decreto, 10/2020). A period of 5 weeks started in which citizens were only allowed to leave their homes for essential work, to buy food and other staple products or for emergencies. On 4th May, citizens were first authorised to leave their homes to exercise or walk, for a maximum of 1 h a day, under strict conditions. From 10th May to 21st June, a progressive de-escalation of confinement measures led to the so-called ‘new normality’ in which Spaniards were allowed to attend their jobs, gather in small groups, and move between provinces as long as they complied with safe distancing and face-covering requirements.

During the first wave of the COVID-19 pandemic, several studies have investigated its mental health consequences in the Spanish adult population (Balanzá-Martínez *et al*., 2020; Garcia-Fernandez *et al*., 2020; Gonzalez-Sanguino *et al*., 2020; Justo-Alonso *et al*., 2020; Pérez *et al*., 2020; Planchuelo-Gomez *et al*., 2020; Cecchini *et al*., 2021; Losada-Baltar *et al*., 2021; Mortier *et al*., 2021; Valiente *et al*., 2021). Overall, these studies have shown a general worsening in mental health throughout the confinement, with prevalence estimates ranging from 9 to 46% among those reporting data on depressive symptoms. Younger age, being female, being a healthcare worker, low income, prior mental disorders, loneliness, and substance use appeared as the strongest factors associated with mental health problems. However, the validity of these findings may be somewhat hindered by at least one of the following drawbacks: (i) non-probabilistic sampling approaches or convenience samples evaluated through online surveys, which increases the risk of selection bias; (ii) cross-sectional design or lack of information on the pre-pandemic period, which does not allow for a proper assessment of the determinants of the observed changes in mental health indicators and (iii) assessment of dimensional measures of psychological distress only.

The study aims to assess whether there is a change in the prevalence of depression and suicidal ideation after the strict lockdown measures during the first wave of the COVID-19 pandemic in Spain; and to assess which are the factors associated with the incidence of a depressive episode or suicidal ideation during the lockdown. Our analysis is based on an adult population-based cohort from the provinces of Madrid and Barcelona, which was evaluated before the pandemic and once again after the COVID-19 lockdown.

## Method

### Sample and recruitment

Non-institutionalised adults (i.e. 18+ years old) from the regions of Madrid and Barcelona participated in this study. These constitute the refreshment sample of the *Edad con Salud* project (ageingandhealth.com) (Miret *et al*., 2014). They were recruited following a multistage stratified design consisting of: (i) a random sample of municipalities (sampling probability proportional to population size); (ii) a random sample of census units from each municipality; (iii) a random sample of households within each census track, and assigned to one of two age groups: 18–49 or 50+ (the second one oversampled). For each household, individuals in the assigned age group were invited to participate; the response rate was 68.0%. Sampling weights were generated for the sample to be representative of the target population, according to the population distribution obtained from the National Institute of Statistics.

Participants were interviewed at their homes between 17 June 2019 and 14 March 2020 (pre-COVID measure). They were reached out again between 21 May 2020 and 30 June 2020 to respond to a telephone interview (post-COVID measure). Trained interviewers conducted the pre- and post-measure interviews, using a Computer-Assisted Personal and Telephonic Interviewing system, respectively. Protocols were approved by the Clinical Research Ethics Review Committees of Parc Sanitari Sant Joan de Déu (Barcelona) and Hospital Universitario La Princesa (Madrid). All participants provided informed consent.

Some participants were unable to respond first-hand due to physical and/or mental limitations, and thus a relative or co-habitant answered in their name. Only first-hand respondents to both interviews were included in these analyses; therefore, out of a sample of 1935 participants, 54 proxy respondents were discarded, making a sample of 1881 participants in the pre-measure. A total of 778 were excluded from the post-measure (81 participants did not provide recontact information, 110 participants could not be contacted, 9 were deceased, 39 were responded by a proxy respondent, 329 either rejected to respond to the post-measure telephone interview or aborted it before finishing and 210 had unspecified incidents), so the final post-measure sample comprised of 1103 participants.

### Measures

Depression was assessed with an adapted version of the Composite International Diagnostic Interview (CIDI; Kessler and Ustün, 2004). An algorithm following the ICD-10 criteria was used to diagnose depression in the previous 12 months (World Health Organization, 1993). For the post-measure interview, an abbreviated version was used, and the items were adapted to ask for a 30-day time span in order to account for an onset while the lockdown measures were in effect. The assessment algorithm in the pre-measure was adapted to use the same item set as in the post-measure. Suicidal ideation comprised a single item asking whether the participant had had suicidal thoughts in the previous 12 months/30 days, for the pre- and post-measure periods, respectively.

The following covariates were also measured: age, sex, education level, whether the participant lived alone (both before and during the lockdown), whether the participant had co-habited/was co-habiting with a relative isolated by COVID-19, whether the participant had been/was concerned about a relative/friend infected by COVID-19, whether the participant had been infected with COVID-19 and its severity, whether the participant had enough quietness at home to get proper rest, whether the household economic situation had worsened due to the COVID-19 emergency, whether the participant had been unemployed due to the COVID-19 emergency, time a day spent in front of screens during the lockdown (working and non-working), pre- and post-measure levels of physical activity according to an abbreviated version of the Global Physical Activity Questionnaire version 2 (GPAQ-2) (Armstrong and Bull, 2006), and the following scales: post-measure score in the Brief Resilience scale (Rodríguez-Rey *et al*., 2016), pre- and post-measures of social support measured with the OSLO3 Social Support scale (Dalgard *et al*., 2006), pre- and post-measures of loneliness measured with the UCLA loneliness scale (Hughes *et al*., 2004), and post-measure of disability assessed with the 12-item World Health Organization Disability Assessment Schedule (WHODAS 2.0) (Luciano *et al*., 2010). The Brief Resilience Scale was taken from the validated version by Rodríguez-Rey *et al*. (2016), whereas the rest of them have been validated in the original in English (as referenced) and were adapted for their use in the Edad con Salud cohort study. All of them had internal consistency indices (i.e. Cronbach's *α*) above 0.70, except for the OSLO3 Social Support scale, which reliability was moderate (*α* = 0.653) and low (*α* = 0.386) in the pre- and post-measures, respectively.

### Data analysis

Sample descriptive statistics were computed for depression, suicidal ideation and all the covariates. Attrition in the pre-measure sample was analysed for differences in sociodemographics and the two outcome variables: sex, depression and suicidal ideation were tested with the *χ*^2^-test; bias-corrected Cramér's *V* (*ϕ*_c_) was computed as a measure of effect size. For age, a two-sample *T*-test was performed, with Hedges' *g* as a measure of effect size.

Prevalence estimates – population-wise and disaggregated by sex and age (grouped in 18–29, 30–49 and 50+ year-olds) – were computed for depression and suicidal ideation in both measures. The differences between both measures were tested with a weighted McNemar's test of symmetry, using the complete data. Bonferroni correction was applied variable-wise to the disaggregated estimates.

To model the risk of incidence after the lockdown, the cases with depression or suicidal ideation in the pre-measure periods were filtered out from the dataset for its corresponding analysis. Then, we performed a weighted logistic regression model on the post-measure. All covariates stated in section ‘Measures’ were initially considered. In the case of suicidal ideation, the pre- and post-measures of depression were also considered as covariates. The following procedures were applied for fitting the models: first, in order to archive better numerical convergence, all interval-level variables were standardised, and categorical covariates that yielded complete separation (Albert and Anderson, 1984) were discarded. Covariates were tested individually with univariate weighted logistic regression models and the Rao and Scott (1984) likelihood-ratio test (without Bonferroni correction, in order to decrease type-II error risk). Among the significant covariates, the ordinal ones were tested for non-linearity with the Wald test, comparing the general model with a model with the linear term only. Whenever the test was non-significant, only the linear term was included. Afterwards, a multivariate weighted logistic model was fit with all the significant covariates. A backward-step procedure was then run, dropping covariates according to the Akaike information criterion statistic. Demographic variables sex and age were fixed, excluding them from dropping. In the model of suicidal ideation, the measures of depression were also fixed. Finally, the resulting model was refit to the subset of complete cases in the covariates selected by the backward-step procedure. As the procedure may select a different subset of covariates for each model, the number of complete cases may also differ.

A significance level of *α* = 0.05 was used throughout. All significance tests were performed applying Bonferroni correction for multiple comparisons (unless stated otherwise). All the analyses were conducted in R v. 4.0.3 (R Core Team, 2019). Package survey v. 4.0 (Lumley, 2004) was used to fit the models.

## Results

### Sample descriptives

Participants with data in both measures differed from the ones excluded in the post-measure in sex ( = 15.80, *p* value <0.001) and age (*t*_1467.34_ = 5.59, *p* value <0.001): the proportion of men excluded (48.8%) was relatively higher than the ones included (39.6%), and the participants excluded were older (mean = 59.6, s.d. = 19.8) than the ones included (mean = 54.8, s.d. = 16.4). However, the effect size was negligible for sex (*ϕ*_c_ = 0.089), and small for age (*g* = 0.270). No significant differences were found in depression between the included and the excluded samples ( = 0.03, *p* value = 0.860, *ϕ*_c_ = 0.000). Regarding suicidal ideation, the excluded sample differed significantly from the included one (0.64 *v*. 2.18%, respectively;  = 7.07, *p* value = 0.008); the effect size was also negligible though (*ϕ*_c_ = 0.052). The descriptive statistics for both outcome variables and the covariates for the sample included in the analysis are shown in Table 1.

**Table 1.** Sociodemographic and health characteristics before and after the confinement

Variable	Pre-confinement		Post-confinement		*p* value*
Age, mean (s.d.)	54.82	(16.35)			
Sex (female), *n* (%)	666	(60.38%)			
Education level, *n* (%)					
Less than primary	97	(8.79%)			
Primary	283	(25.66%)			
Secondary	466	(42.25%)			
Tertiary	257	(23.30%)			
Depression, *n* (%)	99	(8.98%)	87	(7.89%)	0.327
Suicidal ideation, *n* (%)	24	(2.20%)	23	(2.09%)	0.853
Resilience, mean (s.d.)^a^			3.51	(0.63)	
Living alone, *n* (%)	163	(14.78%)	131	(11.88%)	<0.001
Social support, mean (s.d.)^a^	78.34	(17.91)	76.20	(16.41)	<0.001
Loneliness, mean (s.d.)^a^	12.07	(25.13)	12.69	(23.97)	0.489
COVID-19 co-habitant, *n* (%)^b^			43	(3.90%)	
COVID-19 concern, *n* (%)^c^			268	(24.30%)	
COVID-19 infection, *n* (%)^d^					
Not infected			1093	(99.09%)	
Infected			7	(0.63%)	
Infected and hospitalised			3	(0.27%)	
Disability, mean (s.d.)^a^			8.72	(13.43)	
Working screen time (h), mean (s.d.)			3.93	(2.16)	
Non-working screen time (h), mean (s.d.)			1.23	(2.62)	
Home quietness, *n* (%)			1030	(93.64%)	
Economy worsened, *n* (%)			331	(30.15%)	
Unemployed, *n* (%)			179	(16.29%)	
Physical activity, *n* (%)					
Low	353	(32.09%)	910	(82.50%)	<0.001
Moderate	384	(34.91%)	76	(6.89%)	<0.001
High	363	(33.00%)	117	(10.61%)	<0.001

*n*, number of participants; s.d., standard deviation.

* *p* values correspond to a paired-sample *T*-test for the quantitative variables, and a McNemar's test of symmetry for the categorical ones.

a These variables are measured in a 0–100 scale.

b Co-habited/ing with relative isolated by COVID-19.

c Concerned about relative/friend infected by COVID-19.

d Severity of COVID-19 infection.

### Prevalence rates

Estimated prevalence rates are given in Table 2. For depression, it increased from 7.78% in the pre- to 9.82% in the post-measure. According to the McNemar's test, the difference was not significant ( = 1.53, *p* value = 0.216). When considering the differentiated age groups, the difference was more prominent for the 18–29 (increasing from 5.32 to 14.17%) and the 30–49 (increasing from 7.96 to 11.99%) groups, but none of them was significant. However, a significant decrease from 8.48 to 6.41% was observed in the 50+ group ( = 6.46, *p* value = 0.011). For suicidal ideation, the prevalence rate estimate increased from 1.56% in the pre- to 2.78% in the post-measure, but this difference was not significant ( = 1.39, *p* value = 0.239). After Bonferroni correction, none of the disaggregated estimates was significant either.

**Table 2.** Prevalence rate estimates in the pre- and post-measures of depression and suicidal ideation, for the population and disaggregated by sex and group age

	Depression			Suicidal ideation			
Segment	Pre (s.d.)	Post (s.d.)	*p* value	Pre (s.d.)	Post (s.d.)	*p* value
Total	7.78% (0.81%)	9.82% (1.19%)	0.216	1.56% (0.38%)	2.78% (0.66%)	0.239
Sex						
Male	6.28% (1.14%)	8.90% (1.86%)	0.375	1.17% (0.51%)	3.11% (1.14%)	0.110
Female	9.13% (1.13%)	10.54% (1.53%)	0.384	1.91% (0.54%)	2.52% (0.79%)	0.964
Age						
18–29	5.32% (1.88%)	14.17% (4.12%)	0.071	2.21% (1.24%)	4.09% (2.37%)	0.878
30–49	7.96% (1.66%)	11.99% (2.51%)	0.064	0.93% (0.59%)	3.31% (1.39%)	0.018
50+	8.48% (0.86%)	6.41% (0.99%)	0.011	1.85% (0.42%)	1.87% (0.55%)	0.243

s.d., standard deviation.

### Risk of depression after the lockdown

The final regression model for depression was fit with a sample size of 940. Its covariates are given in Table 3, along with their odds ratios (ORs). The coefficient for age was found to be significant, along with the post-measures of Loneliness and Resilience.

**Table 3.** Logistic regression model of depression after the confinement in participants without depression before the confinement

Term	OR	(95% CI)	*z*	*p* value
(Intercept)	0.26	(0.09–0.75)	−2.48	0.013
Age (Pre)	0.97	(0.95–0.99)	−3.17	0.002
Sex	0.74	(0.34–1.63)	−0.75	0.455
Resilience (Post)	0.46	(0.32–0.66)	−4.22	<0.001
Social support (Pre)	0.77	(0.51–1.18)	−1.20	0.229
Loneliness (Post)	1.96	(1.42–2.70)	4.08	<0.001
Disability (Post)	1.26	(0.84–1.91)	1.11	0.269
Working screen time (h)	0.90	(0.80–1.02)	−1.69	0.092
Home quietness	0.42	(0.19–0.90)	−2.22	0.026
Physical activity (Pre)^a^	0.76	(0.49–1.18)	−1.22	0.224

OR, odds ratio; CI, confidence interval; Resilience, Brief Resilience Scale; Social support, OSLO3 Social Support Scale; Loneliness, UCLA Loneliness Scale; Disability, 12-item WHO Disability Assessment Schedule Physical activity (GPAQ-2 abbreviated).

a Included as linear covariate.

The OR for age was 0.971 (*z* = −3.17, *p* value = 0.002); for each year, the risk of developing depression was expected to decrease by 2.9%. For Loneliness (Post), the OR was 1.957 (*z* = 4.08, *p* value <0.001), which means that an increase of 1 standard deviation (s.d.) in the post-measure of the UCLA Loneliness Scale was associated with an increase of 95.7% in the OR of receiving a positive diagnosis of depression in the post-measure. In the case of Resilience (Post), the OR was 0.460 (*z* = −4.22, *p* value <0.001), meaning that an increase of 1 s.d. in the post-measure of the Brief Resilience Scale was associated with a decrease of 54.0% in the OR of receiving a positive diagnosis of depression in the post-measure.

### Risk of suicidal ideation after the lockdown

This model was fit with a sample size of 951; its covariates and their coefficients (as ORs) are shown in Table 4. After Bonferroni correction, the significant covariates were the post-measures of Social support and Resilience. The OR of Social support was 0.352 (*z* = −3.04, *p* value = 0.002). This implies that an increase of 1 s.d. in the post-measure of the Oslo-3 Social Support Scale was associated with a decrease of 64.8% in the OR of reporting having suicidal ideation in the post-measure. The OR for Resilience was 0.334 (*z* = −3.01, *p* value = 0.003), implying a decrease of 66.6% for an increase of 1 s.d. in the post-measure of the Brief Resilience Scale.

**Table 4.** Logistic regression model of suicidal ideation after the confinement in participants without suicidal ideation before the confinement

Term	OR	(95% CI)	*z*	*p* value
(Intercept)	0.00	(0.00–0.02)	−5.60	<0.001
Age (Pre)	0.95	(0.89–1.02)	−1.40	0.161
Sex	0.35	(0.08–1.51)	−1.40	0.161
Depression (Pre)	5.06	(1.01–25.30)	1.98	0.049
Depression (Post)	1.83	(0.27–12.56)	0.62	0.538
Resilience (Post)	0.33	(0.16–0.68)	−3.01	0.003
Social support (Post)	0.35	(0.18–0.69)	−3.04	0.002
Disability (Post)	1.30	(0.86–1.95)	1.25	0.211
Physical activity (Pre) (Ref. Low)				
Moderate	0.45	(0.08–2.39)	−0.94	0.348
High	2.61	(0.76–8.96)	1.52	0.129

OR, odds ratio; CI, confidence interval; Resilience, Brief Resilience Scale; Social support, OSLO3 Social Support Scale; Disability, 12-item WHO Disability Assessment Schedule Physical activity (GPAQ-2 abbreviated).

## Discussion

The current study is the first to assess changes in mental health during the first wave of the COVID-19 pandemic in Spain by using a population-based cohort. Overall, our results did not show significant differences in the prevalence of depression or suicidal ideation from before to after the COVID-19 outbreak. Indeed, the prevalence rate of depression in our study was similar to those reported in other Spanish and European studies in non-epidemic circumstances (Paykel *et al*., 2005; Gutiérrez-Rojas *et al*., 2020). Interestingly, the rates of depression among individuals aged 50+ years showed a significant decrease compared to pre-pandemic. The study findings also found that younger individuals and those feeling loneliness exhibited a significant increase in the risk of developing depression. Resilience showed a protective effect against the risk of depression and suicidal ideation, while individuals perceiving social support were at a lower risk of developing suicidal thoughts.

Among the studies tracking longitudinal changes in mental health from before to during the pandemic, some of them have showed increases in the prevalence rate of depression and suicidal ideation (Daly *et al*., 2020; Niedzwiedz *et al*., 2021; Novotny *et al*., 2020; Pierce *et al*., 2020; Planchuelo-Gomez *et al*., 2020; Winkler *et al*., 2020; McGinty *et al*., 2020*b*) whereas others did not report differences above pre-pandemic levels (Kwong *et al*., 2020; van der Velden *et al*., 2020) or even decreased estimates (van der Velden *et al*., 2021). It is worth noting that all but one of the previous studies measured psychological distress or depressive symptoms. In addition, according to a meta-analysis of longitudinal studies investigating the psychological impact of the COVID-19 pandemic, the initial effect of lockdowns on mental health is relatively small, with no evidence of significant increase in suicide risk (Prati and Mancini, 2021).

The first emotional reactions may represent feelings of fear, anger or sadness in response to an unprecedented situation rather than a mental disorder. More fine-grained analyses have showed that mental health problems remained stable or declined throughout the initial lockdown period (Bryan *et al*., 2020; Chandola *et al*., 2020; Daly *et al*., 2020; Gonzalez-Sanguino *et al*., 2020; Hyland *et al*., 2020; Somma *et al*., 2020; Wang *et al*., 2020; McGinty *et al*., 2020*a*; van der Velden *et al*., 2021), which would be consistent with the notion of a progressive adjustment for managing and overcoming stressful events. Nevertheless, it should be noted that these are findings at a very early stage of the COVID-19 outbreak and different conclusions may hold for the comparisons among rate estimates of mental health conditions in the mid- and long-terms. In this regard, Tanaka and Okamoto (2021) examined whether suicide mortality changed during the pandemic using high-frequency data covering the entire Japanese population. The authors found that there was an initial drop in suicide deaths from February to June 2020, then followed by an increase during the second wave (July to October 2020). Similarly, the Spanish Statistical Office revealed that suicide remained the leading cause of external death during the first months of 2020. However, there was a drop of 8.8% as compared with the same period in 2019 (Spanish Statistical Office, 2021). Initial declines in suicidal behaviours are not unexpected and may be explained by reduced stress derived from workplaces and social interactions, government financial support and limited access to lethal means (Tanaka and Okamoto, 2021).

Specific groups appear to be disproportionately affected by the COVID-19 pandemic. That is the case of young individuals, who may encounter more difficulties coping with certain unexpected life-changing events, consistent with the view of resilience as a life-span process (Portella Fontes and Liberalesso Neri, 2015). In addition, the adverse economic and social consequences of the pandemic might have a greater impact on them (e.g. unemployment, changes in daily routines and social dynamics). Unsurprisingly, the scientific literature has provided broad evidence suggesting a high proportion of individuals with or at higher risk of depressive symptoms or psychological distress during the COVID-19 outbreak within this group (Daly *et al*., 2020; Gonzalez-Sanguino *et al*., 2020; Hyland *et al*., 2020; Kwong *et al*., 2020; Niedzwiedz *et al*., 2021; O'Connor *et al*., 2020; McGinty *et al*., 2020*a*; Valiente *et al*., 2021). Prior studies have repeatedly documented the intimate link between loneliness and depression (van den Brink *et al*., 2018; de la Torre-Luque *et al*., 2019; Lee *et al*., 2021). The consistency of results among other COVID-19-related research is also noteworthy (Chandola *et al*., 2020; Creese *et al*., 2020; Gonzalez-Sanguino *et al*., 2020; Kantor and Kantor, 2020; Novotny *et al*., 2020; Palgi *et al*., 2020; van der Velden *et al*., 2021). Even though little is known yet about the mechanisms underlying this association, there is evidence that loneliness may compromise emotion processing and regulation, can lead to decreased cognitive function, and alter metabolic, endocrine and immune responses (Hawkley and Cacioppo, 2010; Lara *et al*., 2019; de la Torre-Luque *et al*., 2021), all of which have been associated with depression. In our current situation, the risk of loneliness over depression is expected to be heightened. In the opposite corner, the identification of the protective effect of resilience on depression and suicidal ideation accords with recent reports (Killgore *et al*., 2020; Lenzo *et al*., 2020; Novotny *et al*., 2020; Ran *et al*., 2020; Cenat *et al*., 2021). Resilience is the process of effectively coping with uncertainty and hardship. Although this finding may be well-suited for designing interventions to mitigate the risk of depression and suicidal thinking, it remains to be further investigated who are these resilient people and what factors characterise resilience (Huisman *et al*., 2017). Furthermore, social support is among the best well-documented variables to influence suicidal behaviour (Calati *et al*., 2019; Hegerl and Heinz, 2019). Early research has also proposed a similar association between social support and suicidal ideation in the context of COVID-19 (Bryan *et al*., 2020; Fitzpatrick *et al*., 2020; Gratz *et al*., 2020; Papadopoulou *et al*., 2021). For instance, Gratz and colleagues (2020), having analysed data from a nationwide community sample of 500 adults from 45 states, claimed that it is not loneliness but an absence of belongingness and significant connections that accounts for the association of the lockdown to a greater suicide risk. In this sense, Joiner's Interpersonal Theory of Suicide (Joiner *et al*., 2005) proposed that the lack of social connectedness may lead to a potentially lethal suicidal attempt. More recently, Klonsky and May (2015) suggested that there is a three-step process towards suicidal attempts where connectedness protects against the escalation of ideation among individuals suffering both psychological pain and hopelessness.

It will take time to know what the ultimate impact of the COVID-19 outbreak is on mental health. The psychological toll of the pandemic is unquestionable, but the reality is complex. As the pandemic persists, its consequences are predicted to gradually appear, including rising unemployment, financial loss, reduced participation, or inadequate supplies derived from significant cuts in spending on social and health care. The effects on mental conditions are expected to stay and peak later, with variations across populations and nations (Brooks *et al*., 2020; John *et al*., 2020; Ayuso-Mateos *et al*., 2021). Continuous reinforcement of preventive and intervening mental health measures during and in the aftermath of the crisis is thus of global importance. In this regard, a position paper detailed several mental health research priorities in response to the demands of COVID-19 (Holmes *et al*., 2020). These include the collection of high-quality data on the mental health effects of the pandemic across the whole population and vulnerable groups, together with the development, assessment and refinement of driven strategies to address its psychological, social and neuroscientific aspects.

### Strengths and limitations

This research has an important number of strengths. First, the use of an adult population-based cohort following a probabilistic sampling approach. Moreover, this sample comprises subjects of all educational levels and age ranges, as compared to recent published studies that tend to over-represent highly educated people and under-represent the oldest population. Second, this study is one of the few including a baseline evaluation of the participants some months before the pandemic outbreak. Third, data from our study were collected through structured face-to-face home-based interviews and telephone interviews, unlike most prior studies, relying on web-based surveys instead. Fourth, we used a standardised assessment tool providing a clinical diagnosis of major depression, whereas the majority of previous research assessed depressive symptoms through screening tests or non-validated instruments. Finally, we used a large variety of validated instruments and sociodemographic variables to cover a broad-ranging research of potentially vulnerable groups. Our findings need to be also interpreted in the context of its shortcomings. As with all COVID-19-related research, the current study is limited by a short follow-up period, which reduced the power to evaluate the effects of the confinement on depression and suicidal behaviour. However, ours is an ongoing project that will provide information to a more comprehensive understanding of the changes in mental health in the mid- and long-terms. We also acknowledge that some measures were collected retrospectively through self-report, which may be affected by recall or reporting bias, especially for the longer recall period. Finally, as this survey did not intend to generate clinical diagnoses for all mental disorders, some individuals presenting for example bipolar disorder or schizophrenia may have been included in our analytical sample.

## Conclusions

This pandemic has put at the forefront the imperative of taking care for others, particularly among vulnerable groups who are experiencing the most distress. Altogether, our results point to the value of the social factors as strongly associated with mental health conditions, with loneliness and social support maybe representing different risk pathways. Promoting sense of connectedness, experiences of companionship, and meaningful relationships show promise in mental health prevention, especially in times of physical distancing and lockdowns. Future research should strive to evaluate the long-lasting effects of the COVID-19 crisis on mental health.

## Availability of data and materials

Data supporting the findings of this study are available upon a reasonable request.
